# A Highly Sensitive FET-Type Humidity Sensor with Inkjet-Printed Pt-In_2_O_3_ Nanoparticles at Room Temperature

**DOI:** 10.1186/s11671-020-03426-6

**Published:** 2020-10-14

**Authors:** Meile Wu, Zhanyu Wu, Xiaoshi Jin, Jong-Ho Lee

**Affiliations:** 1 School of Information Science and Engineering, Shenyang University of Technology, Shenyang, 110870 China; 2 Huafu High Technology Energy Storage Co., Ltd, Yangzhou, 225600 Jiangsu China; 3 Huafu (JiangSu) Lithium Battery High Technology Co., Ltd, Yangzhou, 225600 Jiangsu China; 4 Department of Electrical and Computer Engineering and Inter-University Semiconductor Research Center, Seoul National University, Seoul, 151-742 Republic of Korea

**Keywords:** Pt-In_2_O_3_, Inkjet printing, Humidity sensor, FET sensor, Work function

## Abstract

In this work, Pt-doped In_2_O_3_ nanoparticles (Pt-In_2_O_3_) were inkjet printed on a FET-type sensor platform that has a floating gate horizontally aligned with a control gate for humidity detection at room temperature. The relative humidity (RH)-sensing behavior of the FET-type sensor was investigated in a range from 3.3 (dry air in the work) to about 18%. A pulsed measurement method was applied to the transient RH-sensing tests of the FET-type sensor to suppress sensor baseline drift. An inkjet-printed Pt-In_2_O_3_ resistive-type sensor was also fabricated on the same wafer for comparison, and it showed no response to low RH levels (below 18%). In contrast, the FET-type sensor presented excellent low humidity sensitivity and fast response (32% of response and 58 s of response time for 18% RH) as it is able to detect the work-function changes of the sensing material induced by the physisorption of water molecules. The sensing mechanism of the FET-type sensor and the principle behind the difference in sensing performance between two types of sensors were explained through the analysis on the adsorption processes of water molecules and energy band diagrams. This research is very useful for the in-depth study of the humidity-sensing behaviors of Pt-In_2_O_3_, and the proposed FET-type humidity sensor could be a potential candidate in the field of real-time gas detection.

## Introduction

Humidity sensors are desired for moisture detection and control in various sectors, such as semiconductor and automotive industries, agriculture, and medical field [1–4]. They can be classified into capacitive type [5–7], resistive type [8–10], solid electrolyte type [11], surface acoustic waves (SAW) type [12], quartz crystal microbalance (QCM) [13], etc. depending on their operation mechanisms and sensing approaches. Among them, resistive-type humidity sensors, which detect the variation in resistivity of the sensing materials with the amount of adsorbed water molecules, have interested researchers particularly because of their simple structure, easy fabrication, and convenient operation and application [14, 15]. In order to develop a reliable resistive-type humidity sensor with high sensitivity and short response and recovery times of resistive-type sensors, numerous novel materials have been investigated [14, 15], and nanostructured metal oxides are identified as strong candidates in consideration of their low cost, high operating stability, and good compatibility [15–19].

Recently, In_2_O_3_, as typical n-type semiconducting metal oxides, has attracted much attention because of its promising sensing characteristics in the detection of various target gasses [20–22]. It was found that the impedance of In_2_O_3_ is sensitive to humidity even at room temperature, especially those doped or decorated with noble metals or other oxides [14, 23–25]. However, those resistive-type humidity sensors based on In_2_O_3_ are mostly evaluated by AC excitation voltage with no DC bias to avoid polarization of the sensors [23]. As a result, the measured current needs to be rehabilitated and rectified to a DC signal for the other scaling or processing [26], which increases the complexity of measurement and limits the application of the sensors. Moreover, most of them present relatively poor resolution and sensitivity for low humidity level detection (lower than 25%) and need further improvement [23, 27].

In this work, a FET sensor platform was fabricated, which has a planner floating gate (FG) facing the control gate (CG) horizontally. Doped In_2_O_3_ nanoparticles with Pt (Pt-In_2_O_3_) were deposited on the FET substrate to serve as the sensing material with inkjet printing process for relative humidity (RH) detection lower than 18%. The special construction of the FET platform makes the deposition of the sensing material very easy and evades the pollution of the channel of the FET substrate. More importantly, unlike the impedance change mechanism of the resistive-type sensor, the FET sensor platform reflects the work function changes of the sensing material, which effectively improves the humidity performance of In_2_O_3_-based sensors. In this article, the RH-sensing performance of the proposed FET-type Pt-In_2_O_3_ humidity sensor was detailedly investigated and compared to a Pt-In_2_O_3_ resistive-type sensor that fabricated on the same silicon wafer. The experiments indicate that the surface work function of Pt-In_2_O_3_ is much more sensitive to the adsorption of water vapor than the resistance change. The mechanism behind the sensing performance of both two sensors and the difference between them were discussed by using energy band diagrams of the sensing material. The adsorption behavior of water vapor on Pt-In_2_O_3_ and the reaction procedures were also explained.

## Methods

### Fabrication of Platforms

To deeply understand the sensing principle of the proposed FET humidity sensor, a resistive-type device with the same Pt-In_2_O_3_ sensing material was also investigated in this paper. The resistive-type (Fig. 1a) and the FET-type sensor platforms (Fig. 1b) were fabricated on the same silicon wafer for a fair comparison between them. Figure 1a presents the empty resistor platform, and the inset is its magnified electrodes after forming the transparent Pt-In_2_O_3_ layer. Figure 1b shows the FET platform proposed in our previous work [28, 29]. It has four electrodes including CG, drain (D), source (S), and body electrodes. To protect the active region of the FET platform as marked in Fig. 1a, an extended FG was adopted, which aligned with the CG in a horizontal direction. Interdigitated structures of the two gates were used for a good capacitive coupling between them. In addition, an SU-8 passivation was also conducted to only expose the sensing region as marked in Fig. 1b and the electrode contact pads. Figure 1 c and d are the schematic cross-sectional views along and perpendicular to the channel of the FET, which are along line A–A’ and line B–B’ in Fig. 1b, respectively. The channel length and width are 2 μm and 2.4 μm, respectively. The main fabrication steps were described as follows. In this work, *p*MOSFET platforms were mainly fabricated as they have lower 1/f noise than the *n*MOSFETs [30]. Firstly, a 550-nm-thick field oxide was grown for the isolation of active regions by local oxidation of silicon (LOCOS) process. A buried channel of the FET was formed by ion implantation, and a 10-nm-thick gate oxide was grown by dry oxidation process at 800 °C. Then, a 350-nm in situ-doped n+ poly-Si layer was deposited and patterned to serve as the FG. The heavily doped p+ source and drain regions were formed by ion implantation process. To prevent the FG and channel from unwanted molecules (for example, H_2_O) and charge traps, an ONO passivation layer consisting of SiO_2_ (10 nm)/Si_3_N_4_ (20 nm)/SiO_2_ (10 nm) was formed on the whole wafer. After defining the contact holes, stacked layers of Cr (30 nm)/Au (50 nm) were deposited consecutively and patterned to serve as the CG, D, S, and body electrodes of FET. Note that the electrodes of the resistive-type sensors were also fabricated simultaneously. Finally, an SU-8 passivation layer formed by spin coating was patterned on top of the platforms by a lithography process to expose only the interdigitated FG-CG area of the FET platform (the sensing region in Fig. 1a), the interdigitated electrode area of the resistor platform, and all pads for the electrode contacts.

**Fig. 1:** The resistive-type and FET-type gas sensors with inkjet-printed Pt-In_2_O_3_ nanoparticles. **a** SEM image of the resistive-type sensor platform. The inset shows magnified electrodes after forming the Pt-In_2_O_3_ sensing layer. **b** SEM image of the FET-type sensor with a FG aligned with a CG horizontally. **c** The schematic cross-sectional view along line A–A’ in **b**. **d** The schematic cross-sectional view along line B–B’ in **b**. The channel length and width are 2 μm and 2.4 μm, respectively

### Materials

In_2_O_3_ nanopowders (≤ 100 nm in diameter), ethanol (99%), 8-Wt% H_2_PtCl_6_ (in H_2_O), and deionized (DI) water were purchased from Sigma-Aldrich (USA) for the preparation of the sensing material. All chemicals in this paper were used without further purification.

### Deposition of Sensing Material

The Pt-In_2_O_3_ sensing material was formed by inkjet printing process. Firstly, In_2_O_3_ nanopowders were dissolved in ethanol and stirred thoroughly to obtain a uniform solution. The 8-Wt% H_2_PtCl_6_ (in H_2_O) solution was further diluted by DI water to the desired concentration and then mixed with the In_2_O_3_ solution together to serve as the precursor ink. The as-prepared ink was printed on both kinds of platforms using an inkjet printer (Omni Jet 100), followed by a 2-h annealing process at 300 °C in air to fully evaporate the solvent from the printed sensing layer. The Wt% of Pt in the sensing layer was just set to be 10 Wt% to focus principally on the analysis of water vapor adsorption effects.

### Measurement Setups

Figure 2 shows the measurement setups used in this work. In Fig. 2, humid gas samples were made by mixing dry air and wet air prepared by injecting dry air through a bubbler, in the mixing chamber. The total flow rate of the humid air sample was fixed at 400 sccm, and the relative humidity was determined by balancing the flow rates of dry and wet air through a multichannel mass flow programmer and calibrated by a humidity calibrator. A reference gas (dry air) with a flow rate of 400 sccm was also used. During the dynamic humidity-sensing test, the reference dry air and the humid air sample were blown to the sensors alternatively. All sensing characteristics of sensors were tested at 25 °C (room temperature). Electrical measurements were carried out by using an Agilent B1500A.

**Fig. 2:** Measurement setups. All characteristics of sensors were tested at 25 °C (room temperature)

## Results and Discussion

Firstly, the basic I-V characteristics of the Pt-In_2_O_3_ resistive-type and FET-type sensors were measured and plotted in Fig. 3 a and b, respectively. Double sweep I-V curve of the resistor shown in Fig. 3a indicates an ohmic contact behavior of the Pt-In_2_O_3_ film to the electrodes in both resistive-type and FET-type sensors. In Fig. 3b, double sweep DC I-V and pulsed I-V (PIV) of the FET-type sensor from positive to negative and back were plotted together for comparison. The inset is the pulse scheme used for PIV measurement. In DC I-V results, hysteresis can be observed, which is induced by charge trapping in the sensing material and at the interface between the sensing material and the ONO passivation stacks. Under the traditional working environment of FET type sensors, DC biases are typically applied to the electrodes for tracing the current sensing signal. However, due to the mentioned charge trapping inside the device, the current of the FET sensor can drift significantly over time, which disturbs the current baseline and degrades the accuracy. In contrast, in PIV of the proposed FET humidity sensor, the hysteresis was restrained by using pulsed gate bias. Upon those results, in order to obtain reliable and stable sensing signals when measuring the transient sensing properties of the FET-type sensor, a pulsed measurement method was adopted [29, 31] which is illustrated in Fig. 4a.

**Fig. 3:** Basic electrical properties of the resistive-type and FET-type Pt-In_2_O_3_ sensors at *T* = 25 °C. **a** Double sweep I-V curve of the resistive-type sensor. The results of forward and reverse voltage sweeps overlap with each other. **b** Double sweep DC and pulsed I-V (PIV) curves of the FET-type sensor. The inset indicates the pulse scheme used for PIV measurement

**Fig. 4:** Sensing performance of two types of sensors for 9.4% RH. **a** Schematic of the FET-type sensor and the pulse scheme used for the measurement of the FET-type sensor in this work. **b** |*I*_D_| of FET-type sensor based on *p*MOSFET decreased obviously as RH increased from 3.3 to 9.4%. The sensor was blown with humid air for 100 s from about 70 to 170 s. **c** DC transient measurement of the resistive-type sensor and no response was observed from the resistive-type sensor for 9.4% RH

Figure 4a shows the pulse scheme and the implementation strategy of the pulsed measurement method for the FET-type humidity sensor. The left side of Fig. 4a is the schematic of the FET-type sensor, and pulsed biases were applied to its CG and D electrodes by two waveform generators of Agilent B1500A. The on time (pulse width) *t*_on_ and off time *t*_off_ in one pulse period were fixed at 20 μs and 1 s, respectively. During the off time *t*_off_, all the CG, D, and S electrodes of the FET were grounded, and no drain current (*I*_D_) was read out. During the on time *t*_on_, appropriate CG and D read voltages (*V*_rCG_ and *V*_rDS_) were applied synchronously to collect *I*_D_ samples. Figure 4 b and c show the sensing behaviors of the FET-type and resistive-type sensors, respectively, upon the exposure to 9.4% relative humidity (RH) for 100 s. Note that, for the resistive-type sensor, only constant DC voltages were adopted. The Pt-In_2_O_3_ resistive-type sensor, which reflects resistance changes of the sensing material, was not sensitive to the increase of RH from 3.3% (dry air) to 9.4%. However, the absolute drain current |*I*_D_| of the *p*MOSFET sensor decreased markedly with the increase of RH and returned back to the original baseline within about 400 s during the recovery period of the sensor. Given that the sensing mechanism of the FET-type sensor is the change in work function of Pt-In_2_O_3_ caused by the adsorption of water molecules, the measurement results indicate that the work function of the sensing material is more sensitive to RH change compared to the resistance. Detailed explanations of this sensing behavior and the reason for the difference in humidity sensitivity between the two platforms were addressed later in this paper.

Next, dynamic response of the FET-type sensor to different RH levels (7.6%, 9.4%, 11.4%, 13.4%, 15.5%, and 17.8%) was measured and is presented in Fig. 5a. The response of the FET-type sensor denoted as *S*_RH_ was expressed by Eq. (1) [32], where *I*_D_D_ and *I*_D_H_ are the original drain current in dry air and the current in a humid environment at a certain RH level, respectively.

1 $$ {S}_{\mathrm{RH}}=\left[\left(\left|{I}_{\mathrm{D}\_\mathrm{D}}\right|-\left|{I}_{\mathrm{D}\_\mathrm{H}}\right|\right)/\left|{I}_{\mathrm{D}\_\mathrm{D}}\right|\right]\times 100\% $$

**Fig. 5:** Humidity detection using the proposed FET-type sensor. **a** Transient humidity sensing measurement at *T* = 25 °C. RH = 3.3%, 7.6%, 9.4%, 11.4%, 13.4%, 15.5%, and 17.8%. **b** *S*_RH_ as a parameter of RH in a range from 3.3 to 17.8%. **c** Variations of *t*_res_ and *t*_rec_ of the FET-type sensor with RH levels

Figure 5b plots the *S*_RH_ as a function of RH ranging from 3.3 (dry air) to about 18%. The *S*_RH_ tends to be proportional to the RH in this range. Note the dynamic response of resistive Pt-In_2_O_3_ sensor to RH was also measured, but no resistance change of the sensing material was observed (from 3.3 to 18% RH). The response time *t*_res_ and recovery time *t*_rec_ are defined as the time required for the current to change to 90% of its final value [33]. Figure 5c presents the variations of *t*_res_ and *t*_rec_ of the FET-type sensor with RH of 3.3–18%. The *t*_res_ reduced slightly with the increase of RH, and all *t*_res_s corresponding to different RH values are less than 60 s. In contrast, the increment in RH has the opposite effect on the *t*_rec_ of the sensor. According to the results, the proposed FET-type humidity sensor has very rapid and high responses to low RH levels at room temperature.

To explain the humidity sensing mechanism of the Pt-In_2_O_3_ FET-type sensor investigated in this paper below about 18% RH, the schematic water molecule adsorption and related energy band diagrams near the interface between ONO stake and sensing material were constructed as shown in Fig. 6. Figure 6a illustrates various kinds of adsorptions of water molecules on the surface of Pt-In_2_O_3_ particles. With the catalytic action of Pt, water molecules are promoted to react with pre-adsorbed oxygen species (${\mathrm{O}}_{\mathrm{ad}}^{-}$) producing hydroxyl groups (–OH) on the surface of In_2_O_3_ as shown in Eq. (2) [34].

2 $$ {\mathrm{H}}_2\mathrm{O}+2\mathrm{In}+{\mathrm{O}}_{\mathrm{ad}}^{-}\longleftrightarrow 2\left(\mathrm{In}-\mathrm{OH}\right)+{\mathrm{e}}^{-} $$

**Fig. 6:** Schematic water molecule adsorption and related energy band diagrams. **a** Chemisorption and physisorption layers of water molecules on Pt-In_2_O_3_ sensing material. **b** The energy band diagram near the interface between the ONO stack and sensing layer before RH detection. It was assumed to be at a flat band state. **c** The energy band diagram after RH detection. Dipoles at the interface decrease the work function of the sensing material

Those hydroxyls leave on the surface of the sensing material and compose the first chemisorption layer because it is difficult to desorb tightly chemisorbed ions at room temperature [35]. Then, during sensing tests, with the increase of RH level, more water molecules start to adsorb on the hydroxyls through double hydrogen bonds and compose the second adsorption layer, which is the first physisorption layer having barely no movable ions inside. When RH level further increases, more layers accumulate after the first physisorption layer filled on the surface of sensing material as shown in Fig. 6a, i.e., the multi-physisorption layers. According to the literatures [23], the impedance of In_2_O_3_ begins to decrease until RH reaches higher than about 54%. At low RH levels, only the first physisorption layer is formed, where there are no movable protons contributing to the electrical conduction. After that, multi-physisorption layers are formed through single hydrogen bonding, where movable protons (H^+^) will be generated by the ionization under an electric field. Those protons hop between the adsorbed water molecules inducing higher conductivity of the sensing material, i.e., the Grotthuss mechanism [27, 36–38]. In this paper, no current change of the Pt-In_2_O_3_ resistive-type sensor was observed, which demonstrates –OH groups have covered the surface of the sensing material and only physical adsorptions of water molecules occurred when RH was increased during the measurements. Consequently, the Pt-In_2_O_3_ resistive-type sensor showed poor sensitivity to RH increments below 18%.

In the case of FET-type sensors, the sensing mechanism is the changes in the work function of sensing material, which is different from resistive-type sensors. According to the results of the resistive-type sensor, under the conditions of RH levels measured in this paper, there is no electron transfer between the sensing material and the water molecules in physisorption layers. However, those adsorbed water molecules can create dipoles at the surface of In_2_O_3_ particles pointing away from the sensing material (Fig. 6a). Figure 6 b and c show the energy band diagram of the In_2_O_3_ near the interface between the sensing layer and the ONO stack before and after moisture detection, which illustrate the effect of the dipoles. From the perspective of energy bands, the chemisorbed hydroxyls have already existed on the surface of the In_2_O_3_ before the test, and we assume that it is at flat band state before moisture detection for convenience (Fig. 6b). The *E*_VAC_, *E*_C_, *E*_F_, and *E*_V_ in the diagrams denote the energy of vacuum, conduction band, valence band, and Fermi level, respectively. The difference between the *E*_VAC_ and *E*_F_ before sensing tests, i.e., the work function, of In_2_O_3_ at the interface between the sensing layer and ONO stack, is defined as *Φ*_S1_. After the physisorption of water molecules, dipoles formed at the interface reduce the electron affinity and result in the uniform decrease of the work function from *Φ*_S1_ to *Φ*_S2_. The difference between *Φ*_S1_ and *Φ*_S2_ is denoted as Δ*Φ* as shown in Fig. 6c. There is barely no electron transfer from physisorbed water molecules to In_2_O_3_. However, the Δ*Φ* can generate electron accumulation in the body of FET near the interface between gate oxide and body, so the |*I*_D_| of *p*MOSFET decreases. In other words, even though there is no change in the resistance of Pt-In_2_O_3_ layer, the dipoles formed by adsorbed water molecules in the physisorption layers can tune the work function of the sensing material and finally induce the drain current changes of the FET-type sensor.

## Conclusions

In summary, a FET-type sensor with inkjet-printed Pt-In_2_O_3_ nanoparticles was investigated for low RH detection ranging from 3.3 to 18% at room temperature. The Pt-In_2_O_3_ resistive-type sensor fabricated on the same silicon wafer was not sensitive to humidity changes at low RH levels. In contrast, the FET-type sensor exhibited fast and excellent humidity response. The principle behind this phenomenon was explained by energy band theory and adsorption behaviors of water molecules on the sensing material. Since only physisorption layers were generated, no electron transfer occurred to contribute to the reduction in resistance of the resistive-type sensor, whereas the physisorbed water molecules formed dipoles that can change the electron affinity and resulted in an increase of work function of the sensing material. Therefore, the proposed FET-type Pt-In_2_O_3_ humidity sensor is promising in the applications of low humidity level detections.

## Data Availability

The datasets used and/or analyzed during the current study are available from the corresponding author on reasonable request.

## Abbreviations

Pt-In_2_O_3_: Pt-doped In_2_O_3_ nanoparticles
FET: Field-effect transistor
RH: Relative humidity
SAW: Surface acoustic waves
QCM: Quartz crystal microbalance
AC: Alternating current
DC: Direct current
FG: Floating gate
CG: Control gate
SU-8: Sukhoi Su-8
MOSFET: Metal-oxide-semiconductor field-effect transistor
LOCOS: Local oxidation of silicon
ONO: Oxide-nitride-oxide stack
D: Drain
S: Source
SEM: Scanning electron microscope
PIV: Pulse I-V
